The article "Exchange Rate Forecasting Based on Deep Learning and NSGA-II Models" was retracted in 2023. Reasons: signs of a paper mill; compromised peer review; unreliable results or conclusions.

# Exchange Rate Forecasting Based on Deep Learning and NSGA-II Models

**DOI:** 10.1155/2021/2993870

**Published:** 2021-09-22

**Authors:** Jun Chen, Chenyang Zhao, Kaikai Liu, Jingjing Liang, Huan Wu, Shiyan Xu

**Affiliations:** SILC Business School, Shanghai University, Shanghai 201800, China

## Abstract

Today, the global exchange market has been the world's largest trading market, whose volume could reach nearly 5.345 trillion US dollars, attracting a large number of investors. Based on the perspective of investors and investment institutions, this paper combines theory with practice and creatively puts forward an innovative model of double objective optimization measurement of exchange forecast analysis portfolio. To be more specific, this paper proposes two algorithms to predict the volatility of exchange, which are deep learning and NSGA-II-based dual-objective measurement optimization algorithms for the exchange investment portfolio. Compared with typical traditional exchange rate prediction algorithms, the deep learning model has more accurate results and the NSGA-II-based model further optimizes the selection of investment portfolios and finally gives investors a more reasonable investment portfolio plan. In summary, the proposal of this article can effectively help investors make better investments and decision-making in the exchange market.

## 1. Introduction

No matter for the purpose of exchange investment or exchange hedging, accurate exchange analysis and forecasting and exchange derivatives trading strategy have become the research contents of institutions and individuals in various countries [1]. A growing number of government agencies, economists, and financial institutions begin to pay attention to the use of financial models to analyze the macro parameters of dynamic time series to predict the exchange rate [2].

However, building a high-precision financial time series prediction model is still a difficult and important topic for scientists, economists, and decision-makers. Traditional methods often fail to capture the complex characteristics of discontinuous, nonlinear, and high frequency in exchange financial time series dataset [3]. In this context, from the perspective of individual or institutional exchange traders, this paper constructs a dual-objective optimization econometric model of exchange forecast analysis portfolio from the whole process of exchange trading platform selection data collection exchange rate analysis exchange portfolio optimization selection, in order to achieve more accurate forecast portfolio selection through technical analysis, the maximization of income and the minimization of portfolio risk [4]. Deep learning has not been widely used in time series prediction, but it has been explored; at present, scholars mainly focus on the time series prediction based on the DBN algorithm, while the time series prediction based on the SRU deep network model is rarely completed [5].

The article "Exchange Rate Forecasting Based on Deep Learning and NSGA-II Models" was retracted in 2023. Reasons: signs of a paper mill; compromised peer review; unreliable results or conclusions.

The rest of the paper is organized as follows: Section 2 is related work on exchange rate forecasting models.  Section 3 contains the design based on the deep learning model, which is described in detail in this paper.  Section 4 contains the results of the deep learning model.  Section 5 concludes some important findings.

## 2. Related Work

For a long time, the study of exchange rate forecasting models has attracted many scientists, economists, and economic policy decision-makers. On the whole, the previous literature mainly explored three areas: first, most studies adopted time-based conditional heteroscedasticity in the standard model and used variability as the main parameter. These models can be classified as the famous ARCH and GARCH methods first proposed by Ayachi et al. [6]. This type of model describes the evolution of the importance of uncertainty and also shows the time evolution of the average square error. Although the ARCH and GARCH frameworks have been proven to be very effective in predicting volatility changes, the academic circles have not been able to unify the economic explanations for the final clustering of uncertainty. Therefore, in [7], the variability equivalent to a one-year period is very predictable, but in [8], as well as [9], all of the research results confirmed that the predictability of volatility mainly exists in a short-term dimension. In addition, it is further proposed that the effectiveness of the model based on ARCH evaluation is also significantly affected by structural changes. Secondly, another type of exchange rate forecasting model attempts to establish a reasonable expectation hypothesis by rationally analyzing the characteristics of macro fundamentals and further constructs an exchange rate forecasting model [10]. These models are often based on the analysis of the domestic currency and the supply and demand of a currency. The longest cited analysis indicators generally include relative inflation rate, relative basic interest rate, gross domestic product, trade balance, income level, and other parameters [11]. In a nutshell, this type of forecasting model is generally based on an average purchasing power model, a covered or noncovered interest rate evaluation model, and a currency model. However, this type of forecasting model based on macro fundamental analysis also exposes a series of shortcomings and deficiencies. For example, policy factors in various countries and changes in investor psychology often lead to unpredictable black-market speculation, or different influencing factors often occur in different periods, producing a variety of impact results [13]. Therefore, in [14], it is pointed out that the predictive ability of this kind of structured model in the short term cannot even be a pure random walk model. As deep learning returns to the mainstream of research and attracts more and more attention from researchers, deep learning algorithms have also completed the exploration of empirical applications in many fields, including time series forecasting [15]. Yao et al. proposed a DBN model composed of a multilayer strict Bozeman machine for time series forecasting [16]. This model uses ATS benchmark data and the particle swarm optimization algorithm. In this research, the DBN algorithm has been proved to successfully surpass the traditional MP neural network model and statistical model ARIMA. Hu et al. proposed a method based on deep learning, and the integrated algorithm of the DBN model is used for time series forecasting [17]. Peng et al. proposed a deep structure based on DBN model multitask learning for traffic flow forecasting [18]. In addition, Prusa and Khoshgoftaar used the training set to construct an overcomplete dictionary and proposed a time series prediction based on sparse coding [19]. Parwez et al. used the sparse coding model to expand the method of online time series prediction and solved the L1-standard convex optimization problem for each new time series vector [20]. Finally, nowadays, more and more exchange forecasting model researchers have begun to shift their thinking to the field of artificial intelligence. Most of this type of research results use time series statistics to predict the movement of currency exchange rates, and it has gradually been proved to greatly surpass traditional predictions. Method [21]: this type of forecasting method mainly includes regression models and agency models based on the concept of behavioral finance and genetic algorithms and artificial neural network models; these models often fall into the trap of local minimums [22]. In addition to supporting vector regression, the SVR model is considered to be a stronger prediction method than the ANN model because it can achieve global optimization [23]. All in all, among a large number of parameter statistical models, ANN has the advantage of being less affected by its model misidentification problem, and it is the most used predictive model so far [24]. After years of improvement and optimization, although significant improvements have been achieved in the accuracy of the model, it still cannot surpass the maximum hidden layer setting of 2 layers due to the problem of nonconvex optimization. Therefore, the difficulty of using deep networks to improve accuracy has been unable to move forward [25–30].

The article "Exchange Rate Forecasting Based on Deep Learning and NSGA-II Models" was retracted in 2023. Reasons: signs of a paper mill; compromised peer review; unreliable results or conclusions.

This article combines theory with practice and innovatively proposes an innovative model of dual-objective optimization measurement for exchange rate forecasting and analysis of investment portfolio. On the whole, the dual-objective optimization measurement model of exchange forecasting and analysis investment portfolio proposed in this paper proposes a selection of data collection from exchange trading platforms, which has a strong reference and guiding significance for the practical application of exchange investors. Specifically, the significance of the two core algorithms proposed by the model is as follows: the exchange rate prediction algorithm based on SRU deep learning obtains more accurate results than typical traditional exchange rate prediction algorithms (such as neural networks and support vector machines); the dual-objective measurement optimization algorithm of the investment portfolio further uses the results predicted by the above model to optimize the selection of investment portfolios and finally gives investors a more reasonable investment portfolio plan.

## 3. Exchange Rate Forecast Analysis and Portfolio Optimization Econometric Model Design Based on Deep Learning

### 3.1. Deep Learning Model

Taking a typical single output neural network as an example, Figure 1 shows a neural network with three input units, three hidden units, and one output unit.

The parameter of the neural network is defined as (*W*, *b*)=(*W*^(1)^, *b*^(1)^, *W*^(2)^, *b*^(2)^), where *W*^(1)^ represents the parameter connecting the j-th element of layer *L* and the first element of layer *L* + 1, and *b*^(1)^ represents the deviation of the i-th element of layer *L* + 1. Therefore, in the neural network structure shown in Figure 1, *W*^(1)^ ∈ *ℜ*^3×3^, *W*^(2)^ ∈ *ℜ*^3×3^; in addition, the parameter *W*^(1)^ ∈ *ℜ*^3×3^ is defined as the activation factor of the i-th unit of layer *L*, which can also be understood as the output of the neural unit, and the output of layer L3 is defined as *h*_*w*,*b*(*x*)_. In the structure shown in Figure 1, the data parameter is a numerical value. So far, the structure function relationship of the neural network can be expressed as in the following formulas:

(1) $$\begin{array}{c} a_{i}^{\left(1\right)}=f\left(w_{11}^{\left(1\right)}\chi_{1}+w_{12}^{\left(1\right)}\chi_{2}+w_{13}^{\left(1\right)}\chi_{3}+b_{1}^{\left(1\right)}\right),\\ a_{2}^{\left(2\right)}=f\left(w_{21}^{\left(1\right)}\chi_{1}+w_{22}^{\left(1\right)}\chi_{2}+w_{23}^{\left(1\right)}\chi_{3}+b_{2}^{\left(1\right)}\right),\\ a_{3}^{\left(2\right)}=f\left(w_{31}^{\left(1\right)}\chi_{1}+w_{32}^{\left(1\right)}\chi_{2}+w_{33}^{\left(1\right)}\chi_{3}+b_{3}^{\left(1\right)}\right),\\ h_{wb}\left(x\right)=a_{1}^{\left(3\right)}=f\left(w_{11}^{\left(2\right)}a_{1}^{\left(2\right)}+w_{12}^{\left(2\right)}a_{2}^{\left(2\right)}+w_{13}^{\left(2\right)}a_{3}^{\left(2\right)}+b_{1}^{\left(2\right)}\right). \end{array}$$

Generally, there are two choices in a neural network; one is sigmoid function:

(2) $$\begin{array}{c} f\left(z\right)=\frac{1}{1+\exp\left(-z\right)}. \end{array}$$

Another commonly used activation function is the hyperbolic tangent function (tanh function):

(3) $$\begin{array}{c} f\left(z\right)=\tanh\left(z\right)=\frac{e^{z}-e^{-z}}{e^{z}+e^{-z}}. \end{array}$$

Take a typical small single output neural network as an example, as shown in Figure 2: Layer I1 is the input layer (Input), Layer L3 is the output layer (Output), and Layer L2 is the hidden layer because its neurons cannot be observed. As shown in Figure 2, the neuron marked with +1 is a deviation unit, which is equivalent to an intercept term. All in all, this is a neural network with three input units, three hidden units, and one output unit.

The article "Exchange Rate Forecasting Based on Deep Learning and NSGA-II Models" was retracted in 2023. Reasons: signs of a paper mill; compromised peer review; unreliable results or conclusions.

When the network structure is more complex, in order to make the structure function more concise and clear, the weighted sum of the input parameters of the i-th unit of layer *L* is defined as *z*_i_^*l*^ and then *z*_i_^(2)^=∑_*j*=1_^*n*^*W*_*ij*_^(1)^*x*_*j*_+*b*_*i*_^(*l*)^; therefore, *a*_*i*_^(*l*)^=*f*(*z*_i_^(*l*)^)*s*. The structure of the neural network is written as a more concise function, which is as follows:

(4) $$\begin{array}{c} z^{\left(2\right)}=W^{\left(1\right)}x+b^{\left(1\right)}, \end{array}$$

(5) $$\begin{array}{c} a^{\left(2\right)}=f\left(z^{\left(2\right)}\right), \end{array}$$

(6) $$\begin{array}{c} z^{\left(3\right)}=W^{\left(2\right)}a^{\left(2\right)}+b^{\left(2\right)}, \end{array}$$

(7) $$\begin{array}{c} h_{w,b}\left(x\right)=a^{\left(3\right)}=f\left(z^{\left(3\right)}\right). \end{array}$$

This article will use the deep learning algorithm that has good performance in extracting dataset features, and the SAE-SVR algorithm is integrated to enhance its prediction ability. Therefore, this paper finally proposes an innovative integration algorithm for a more accurate prediction of time series. The following will be the introduction of the innovative deep learning algorithm based on SAE-SVR.

Its structure is shown in Figure 3. The neural network structure discussed before is often based on the situation that the number of hidden layer units S2 of L2 layer is small, but when the number of hidden layer units is large (even far larger than the number of input), it can still get better performance by imposing hidden layer restrictions.

The article "Exchange Rate Forecasting Based on Deep Learning and NSGA-II Models" was retracted in 2023. Reasons: signs of a paper mill; compromised peer review; unreliable results or conclusions.

Specifically, this paper constructs a system with an input layer, an output layer, and K hidden layers of the deep neural network; each layer is composed of sparse coding. The whole process can be divided into six steps as shown in Figure 3.

### 3.2. Exchange Rate Forecast Analysis and Portfolio Optimization

From the perspective of individual or institutional investors in exchange trading, this paper explores the core process of exchange data analysis and portfolio measurement and selection in the process of exchange derivatives trading and investment. In the past, exchange-related research only focused on the research of exchange influencing factors, exchange determinant model, exchange rate forecast, and other fields. Standing in the whole process of exchange investment and trading, they generally showed the characteristics of a single link. The authors of this paper propose an overall framework of exchange derivatives investment analysis trading, as shown in Figure 4.

For a diversified exchange portfolio, the fundamental purpose of portfolio selection among different exchange currency pairs is to maximize the return and minimize the risk. For the diversified exchange portfolio involved in this paper, the return vector of N assets is set as *R* = (*R, R, RZ*), which skillfully represents the proportion of investment and the *i*-th exchange asset. The expected return of the portfolio is expressed as *Er* (*x*); the risk of the portfolio is expressed as *IR (x)*; *con (R, R)* is the covariance of the i-th exchange rate and the *j*-th exchange rate; and then the double objective measurement model of exchange portfolio is established as follows:

(8) $$\begin{array}{c} \max\;\text{ER}=\overset{N}{\underset{i=1}{\sum }}x_{i}R_{i}\\ \min\;\text{VR}\left(\lambda \right)=\overset{i^{\nu }}{\underset{i=1}{\sum }}x_{i}\text{std}\left(R_{i}\right)\\ \text{s.t.}\;\overset{N}{\underset{i=1}{\sum }}x_{i}=1,\;x_{i}\geq 0,i=1,2,\ldots ,N,N=28. \end{array}$$

Under the condition that the expected return rate ER (*R*) is the largest and the risk VR (*R*) of the portfolio is the smallest, the investment allocation scheme of the portfolio is obtained. In the process of realizing the dual-objective measurement model of diversified exchange portfolio for 28 currency pairs, this paper adopts NSGA-II, which is a fast nondominated sorting genetic algorithm model with an elitist strategy proposed by Kalyanmoy Deb. NSGA-II is an improvement on the NSGA algorithm. The NSGA algorithm is a genetic algorithm based on Pareto sorting, which can directly solve multiobjective optimization problems. Each time, it can get a different set of noninferior solutions. The innovation of NSGA-II lies in the hierarchical design of noninferior sorting algorithm and the crowding distance, which can find a good Pareto optimal solution, quickly approach the Pareto frontier, and greatly improve the performance of the NSGA algorithm.

The article "Exchange Rate Forecasting Based on Deep Learning and NSGA-II Models" was retracted in 2023. Reasons: signs of a paper mill; compromised peer review; unreliable results or conclusions.

Specifically, the flow of the two-objective measurement optimization algorithm based on NSGA-II is shown in Figure 5. In the NSGA-II algorithm, the three core steps are as follows:

Step 1: design of the fast nondominant sorting operator.
The key to designing a multiobjective optimization problem is to find Pareto optimal solution set. The fast nondominant ordering in the NSGA-II algorithm is to layer the population according to the level of noninferior solution, and its function is to guide the search to Pareto optimal solution set direction. It is a cyclic adaptive value grading process. Firstly, the nondominant solution set in the group is found, and the first nondominant layer *f* is identified. All the individuals are given (where I is the nondominant order value of individual I) and are removed from the whole group: then, the nondominant solution set in the remaining group is found, the second nondominant layer F2 is recorded, and the individual is given. This is done until the whole population is stratified, and the individuals within the same layer have the same nondominant order *m*∗.
Step 2: the design of the individual crowding distance operator.
In order to be able to sort selectively within individuals, NSGA-II proposes the concept of individual crowding distance. The crowding distance of individual I is the distance between the two individuals *I* + 1 and *I* − 1 adjacent to *I* in the target space. The calculation steps are as follows:
   
*I*. Initialize the distance for the same layer individual. Make l[l] = 0 (where l[l] represents the crowded distance of any individual I).
   
*II*. The individuals in the same layer are arranged in ascending order of the m-objective function value.
   
*III*. Make the individuals on the sorting edge have the choice advantage. Given a large number W, make *z*[0] = *z*[i] = 0.
   
*IV*. For individuals in the middle of the order, the crowding distance is calculated.
   
*V*. For different objective functions, repeat steps II–IV to get the crowding distance 4L of individual I. by selecting the individuals with large crowding distance as a priority, the results can be distributed evenly in the target space to maintain the diversity of the population.
Step 3: the design of elite strategy selection operator.
Elite strategy is to keep the excellent individuals in the parent generation directly into the offspring, so as to prevent the loss of Pareto optimal solution. The elite strategy selection operator is divided into three indexes by the parent *C*, *P*, the offspring *P*, and the synthetic population *R*. The optimal selection was carried out to form a new parent population *C*. Finally, the order of filling *C* from large to small is continued according to the crowd distance of individuals in *Fi* until the population number reaches *N*.

The article "Exchange Rate Forecasting Based on Deep Learning and NSGA-II Models" was retracted in 2023. Reasons: signs of a paper mill; compromised peer review; unreliable results or conclusions.

## 4. Model Evaluation Results

### 4.1. Evaluation Standard of the Econometric Model

Referring to the evaluation of the traditional time prediction model, this paper uses three statistical parameters: mean absolute error, mean square error, and root mean square error as the standard to evaluate the effectiveness and accuracy of the integration algorithm proposed in this paper. The specific calculation method is as follows:

(9) $$\begin{array}{c} \text{MAE}=\sum_{i=1}^{n}\frac{|{\overset{\wedge }{y}}_{l}-y_{i}|}{n},\\ \text{MSE}=\sum_{i=1}^{n}\frac{{\left(y_{l}-y_{i}\right)}^{2}}{n},\\ \text{RMSE}=\sqrt{\sum_{i=1}^{n}\frac{{\left(y_{l}-y_{i}\right)}^{2}}{n}}. \end{array}$$

### 4.2. Empirical Results of the Artificial Neural Network Model

In this paper, the time series toolbox of the MATLAB r2o15a system is used for the study using the proposed model. In this part, the EURUSD dataset is taken as an example.

First of all, data conversion should be carried out according to the data format required by the MATLAB time series toolbox. The algorithm is as follows:

  Step 1: import the exchangeate.xlsx file containing the time series information of 28 currencies to the MATLAB workspace.
  Step 2: extract the 1eurusd dataset in exchangerate.xlsx, which is in the double storage format.
  Step 3: create an empty cell array with the same size as the 1eurusd dataset.
  Step 4: use the loop statement to store the double data of 1eurusd in the cell array.
  Step 5: save the cell array in .Mat format to bin file, and name it 1eurusd. Mat.

After dealing with the dataset format in accordance with Ann toolbox, the toolbox based on MATLAB r2015a can choose the visual toolbox or the algorithm based on *M* code. Firstly, this paper uses visualization tools to carry out 1eurusd data training and testing process; the specific process is as follows.

First of all, based on the characteristics of financial time series, this paper selects the NAR structure network, that is, the model of nonlinear autoregressive, for empirical study.

Secondly, the training set, validation set, and testing set of the whole EURUSD dataset are divided into 70%, 20%, and 10%. Among them, the training set is used to train the neural network step by step, in order to maximize the network parameters in line with the characteristics of the dataset, but if the training is excessive, it will produce an overfitting phenomenon, so the validation set is used to judge and prevent the neural network from overtraining. After the training set and validation set, the neural network gets a fixed parameter which will not change. The testing set uses it to evaluate the performance of network training.

The article "Exchange Rate Forecasting Based on Deep Learning and NSGA-II Models" was retracted in 2023. Reasons: signs of a paper mill; compromised peer review; unreliable results or conclusions.

Thirdly, we need to set the network structure, and temporarily determine that the hidden layer element is 10 and the lag window is 6. Because the neural network debugging is a process of feedback and adjustment according to the training results, the subsequent empirical study will continue to adjust the number of hidden layer units and lag window until it meets the standard.

The training effect of the neural network is mainly determined by two parameters. They are error autocorrelation and time series response, respectively. The performance of the neural network is judged according to the performance of the error values displayed by these two parameters. It can be judged from Figures 6 and 7 that the autocorrelation error of the error autocorrelation is within the confidence interval, and the error between the predicted value and the actual value is also around 0, so the proposed model performs well.

Further investigation of its MSE value shows that, as shown in Figure 8, the best MSE result of its validation set is 2.2106 × 10^−4^.

However, considering that the implementation of the deep learning algorithm of graphic visualization is intuitive and easy to understand, it has a large limitation and not strong extension, which cannot fully meet the needs of this experiment. Therefore, this paper also improves the algorithm code of the deep learning model.

### 4.3. Empirical Results of the Support Vector Regression Model

The STR model algorithm used in this paper adopts the libswm version 3.21 toolbox jointly developed by Chih Chung Chang and Chih Jen Lin and updated in December 2015. In the specific empirical process, we still need to preprocess the data first. Taking the EURUSD dataset as an example, the SVM type selected in this paper is Nu SVR, and the radial basis kernel function, namely, *e*^*∗*^, is used. The gamma value set in this paper is 0.06. According to the above process, this paper further makes an empirical calculation on 28 currency pair datasets, and the results are summarized in Table 1.

## 5. Empirical Results of Exchange Portfolio Based on Deep Learning

Based on deep learning, the dual-objective measurement model of the exchange portfolio is realized by using the MATLAB platform. In the specific operation, this paper uses gamultiobj function included in the genetic algorithm and direct search toolbox to complete.

The article "Exchange Rate Forecasting Based on Deep Learning and NSGA-II Models" was retracted in 2023. Reasons: signs of a paper mill; compromised peer review; unreliable results or conclusions.

The input data of this algorithm comes from the prediction results of the SAE-SVR integrated model output in the previous process. Because of the normalization pretreatment of data before training the model, it is necessary to restore the data before completing the algorithm. The restoration algorithm is as follows:

(10) $$\begin{array}{c} S_{i}=S_{\max}-Z_{i}\left(S_{\max}-S_{\min}\right). \end{array}$$

*Z*_*i*_ represents the data after normalization pretreatment, *S*_*i*_ represents the data after restoration, and the restored output dataset is obtained. This paper takes the Forex data of the 50 days before June 1, 2021, as an example, according to formulas (11) and (12) of the dual-objective econometric model of Forex portfolio designed in this paper:

(11) $$\begin{array}{c} \max\text{ER}\left(x\right)=\sum_{i=1}^{N}x_{i}R_{i}, \end{array}$$

(12) $$\begin{array}{c} \min\text{VR}\left(x\right)=\sum_{i=1}^{N}x_{i}\text{std}\left(R_{i}\right), \end{array}$$

(13) $$\begin{array}{c} \text{s.t.}\sum_{i=1}^{N}x_{i}=1,\;x_{i}\geq 0,i=1,2,\ldots ,N,N=28. \end{array}$$

Based on MATLAB, the NSGA-II exchange portfolio double objective measurement optimization algorithm is realized, and the optimal portfolio solution with 28 currency pairs as investment targets is calculated. In order to approach Pareto point more accurately and quickly, this paper first considers that 13 currency pairs with negative return rates are cut. Only the remaining 15 currency pairs are counted.

The Pareto points obtained from the experimental results are shown in Figure 9. This paper verifies the different results of the algorithm under different iterations. The repeated experimental results show that the algorithm has the highest expected rate of return and the lowest investment risk under 150 iterations.  Table 2 shows nine investment portfolio schemes under 150 iterations; the order of the expected return is from large to small:

It can be seen from the experimental results that the proportion of exchange asset investment with negative forecast return is 0, which is in line with the actual requirements. According to the results of the portfolio, different investors can choose the corresponding portfolio according to their own characteristics. For risk averse investors, option 9 can be chosen. Although the expected rate of return is only 0.919%, the risk is relatively low, only 0.006224. On the contrary, for investors who have higher requirements for return and can bear certain risks, option 1 can be selected. At this time, the expected return rate is 1.6%, but the risk is also relatively high, and they have to bear 0.009088. Compared with the solution of linear programming, the expected rate of return has been improved and the diversity of investment is also reduced, so the quality of portfolio has been significantly improved. It has a good reference value in the practical operation of investors.

The article "Exchange Rate Forecasting Based on Deep Learning and NSGA-II Models" was retracted in 2023. Reasons: signs of a paper mill; compromised peer review; unreliable results or conclusions.

### 5.1. Experimental Results and Comparisons

The experiment summarizes the exchange rate prediction results based on the deep learning algorithm. Through the comparison in Table 3, it can be seen that the MSE prediction accuracy of the deep learning algorithm can reach four digits after the decimal point, while the MSE prediction accuracy of the SVR algorithm can only reach three digits after the decimal point. It can be seen that the performance of the deep learning algorithm in exchange rate prediction is obviously better than the SVR algorithm. In this paper, the lifting value of SAE-SVR compared with deep learning algorithm is defined as follows:

(14) $$\begin{array}{c} \text{promoted}=\frac{|\left(\text{SAESVR}\right)\text{MSE}-\left(\text{ANN}\right)\text{MSE}|}{\left(\text{ANN}\right)\text{MSE}|}. \end{array}$$

According to the calculation results of the lifting column, the lifting values of 28 currency pairs are negative except for euro against US dollar, 5usdcad, 7gbpcad, 10gbpaud, 11usdjpy, 22usdcny, 23eurcny, 25cadcny, and 26audcny; that is, the prediction results of deep learning algorithm are better than the SAE-SVR algorithm proposed in this paper, and the lifting values of other 19 currencies are positive, which means that SAE-SVR algorithm has good prediction accuracy. The reason may be that too many datasets lead to certain errors, or the accuracy of the deep learning prediction algorithm proposed by this problem needs to be further improved, which will be gradually improved in future research. In this case, in order to further verify the prediction optimization degree of the SAE-SVR algorithm, add the promotion values of 28 currency pairs, and the total values of MSE and MAE are 610.92% and 240.61%, respectively. In other words, the SAE-SVR algorithm is 6 times higher than the deep learning algorithm in exchange rate prediction based on MSE. In short, the deep learning algorithm proposed in this paper has better performance than the traditional algorithm.

## 6. Conclusion

Deep learning uses the current cell data and the point-by-point product calculation method for learning. Its structure can be achieved through simple units. Form superposition construction, while using the jump connection method to prevent overfitting and the disappearance of gradient problems, significantly improving the learning speed and prediction accuracy of the deep network. Specifically, the two core algorithms proposed in the model, SVR exchange rate forecasting algorithm based on deep learning of stacked autoencoders, achieve more accurate results than the neural network and support vector machine. The dual-objective econometric optimization algorithm based on NSGA-II further applies the prediction results of the SAE-SVR integrated model to portfolio selection optimization and finally gives investors a more reasonable portfolio plan. Investors can operate in the market directly according to the results of this algorithm by using appropriate exchange derivatives tools. In terms of data selection, this paper uses the effective historical data of Metatrader4 real exchange trading platform and the direct safe exchange rate to currency provided by SAFE and selects a total of 52223 real data of 28 currency pairs from March 23, 2009, to February 1, 2016. This paper uses the MATLAB R2015a experimental platform under the 32-bit Windows 7 operating system. Finally, the innovation model proposed in this paper is realized by self-programming, and the ideal results are achieved. On the one hand, this paper can try more algorithms in deep learning. In addition to stack autoencoders, the typical algorithms of deep learning also include deep belief networks and convolutional neural network. In the next step, we should combine these two deep learning algorithms to do more research and empirical research on exchange forecasting algorithms. On the other hand, this paper only studies the technical aspects of exchange rate analysis, but the analysis of fundamentals is only limited to the carding and elaboration of the influencing factors of macro fundamentals, but there is no further research on the effect of the correlation of the influencing factors. This point can also be used as the next research direction of this paper.

The article "Exchange Rate Forecasting Based on Deep Learning and NSGA-II Models" was retracted in 2023. Reasons: signs of a paper mill; compromised peer review; unreliable results or conclusions.

## Figures and Tables

**Figure 1:** Single output small neural network structure diagram.

**Figure 2:** Distribution of deep learning algorithm integrated by SAE-SVR. (a) Process 1. (b) Process 2. (c) Process 3. (d) Process 4. (e) Process K.

**Figure 3:** The integrated model structure of deep learning algorithm based on SAE-SVR integration.

**Figure 4:** Forex Analysis: the overall framework of the trading model.

**Figure 5:** NSGA-II-based forex portfolio dual-objective metering optimization algorithm process.

**Figure 6:** Correlation results for the proposed model.

**Figure 7:** Time series response results for the proposed model.

**Figure 8:** Prediction of the MSE value of the model based on deep learning.

**Figure 9:** Model Pareto points set for different iterations. (a) 50 iterations. (b) 100 iterations. (c) 150 iterations. (d) 200 iterations. (e) 300 iterations.

**Table 1:** Empirical regression test results of 28 currency pairs dataset SVR.

Dataset	MSE	MAE	RMSE
1EURUSD	0.0026098	0.0399	0.051087
2GBPUSD	0.0011528	0.0272	0.033954
3AUDUSD	0.0003145	0.0143	0.017735
4EURGBP	0.0015129	0.0307	0.038896
5USDCAD	0.0022363	0.0332	0.04729
6EURCAD	0.0005757	0.0189	0.023995
7GBPCAD	0.0007986	0.0215	0.028259
8AUDCAD	0.00068021	0.0198	0.02608
9EURAUD	0.00024962	0.0114	0.015799
10GBPAUD	0.00062255	0.0191	0.024951
11USDJPY	0.00465398	0.0567	0.06822
12EURJPY	0.00034466	0.0142	0.018565
13GBPJPY	0.00141236	0.0299	0.037581
14CADJPY	0.00055366	0.0177	0.02353
15AUDJPY	0.0002919	0.0129	0.017087
16USDCHF	0.0009669	0.0154	0.031095
17EURCHF	0.0022557	0.0304	0.047494
18GBPCHF	0.0010526	0.0155	0.032444
19CADCHF	0.00111476	0.0208	0.033388
20AUDCHF	0.0015979	0.0268	0.039974
21CHFJPY	0.0014423	0.0224	0.037978
22USDCNY	0.00103769	0.0135	0.032213
23EURCNY	0.0017301	0.0318	0.041594
24GBPCNY	0.00052641	0.0163	0.022943
25CADCNY	0.0045405	0.0536	0.067383
26AUDCNY	0.00255696	0.0403	0.050566
27JPYCNY	0.00255696	0.0349	0.042356
28CHFCNY	0.0316333	0.1728	0.177857

**Table 2:** Forex portfolio scenarios based on NSGA-II algorithms.

Portfolio options	EUR USD	GBP USD	AUD USD	EUR GBP	USD CAD	EUR CAD	GBP CAD	AUD CAD	EUR AUD	GBP AUD
1	0	0	3.75%	0	0	0	0	0	0	0
2	0	0	3.59%	0	0	0	0	0	0	0
3	0	0	3.36%	0	0	0	0	0	0	0
4	0	0	3.34%	0	0	0	0	0	0	0
5	0	0	3.25%	0	0	0	0	0	0	0
6	0	0	3.08%	0	0	0	0	0	0	0
7	0	0	2.85%	0	0	0	0	0	0	0
8	0	0	2.80%	0	0	0	0	0	0	0
9	0	0	2.76%	0	0	0	0	0	0	0

Portfolio options	USD JPY	EUR JPY	GBP JPY	CAD JPY	AUD JPY	USD CHF	EUR CHF	GBP CHF	CAD CHF	AUD CHF

1	5.15%	0.01%	0.28%	78.50%	0.52%	3.63%	0	0.87%	1.85%	0.20%
2	6.32%	0.07%	0.28%	69.01%	0.73%	3.77%	0	1.26%	1.65%	0.25%
3	7.66%	0.18%	0.25%	54.07%	4.75%	3.93%	0	1.87%	1.34%	0.32%
4	7.82%	0.19%	0.25%	52.90%	4.68%	3.95%	0	1.92%	1.31%	0.33%
5	7.31%	0.21%	0.27%	49.77%	0.97%	4.05%	0	2.08%	1.22%	0.33%
6	6.70%	0.26%	0.25%	39.07%	1.04%	4.20%	0	2.53%	0.96%	0.36%
7	11.79%	0.41%	0.25%	27.71%	1.26%	4.34%	0	2.97%	0.84%	0.48%
8	11.04%	0.41%	0.24%	22.68%	5.27%	4.38%	0	3.27%	0.67%	0.48%
9	12.13%	0.44%	0.26%	22.63%	1.33%	4.43%	0	3.18%	0.73%	0.50%

Portfolio options	CHF JPY	USD CNY	EUR CNY	GBP CNY	CAD CNY	AUD CNY	JPY CNY	CHF CNY	ER(X)	SD(X)

1	0.16%	0	2.23%	1.85%	0.53%	0.57%	0	0	0.016146	0.009088
2	0.24%	0	2.26%	2.62%	7.35%	0.70%	0	0	0.014967	0.008605
3	0.43%	0	2.37%	3.45%	15.21%	0.90%	0	0	0.013532	0.008071
4	0.44%	0	2.37%	3.55%	16.12%	0.92%	0	0	0.013375	0.008005
5	0.40%	0	2.32%	3.84%	23.09%	0.97%	0	0	0.012356	0.007590
6	0.46%	0	2.34%	3.70%	34.03%	1.10%	0	0	0.010708	0.006995
7	0.67%	0	2.40%	6.37%	36.42%	1.27%	0	0	0.009864	0.006491
8	0.71%	0	2.47%	5.97%	38.32%	1.34%	0	0	0.009543	0.006455
9	0.67%	0	2.41%	6.86%	40.33%	1.34%	0	0	0.009190	0.006224

The article "Exchange Rate Forecasting Based on Deep Learning and NSGA-II Models" was retracted in 2023. Reasons: signs of a paper mill; compromised peer review; unreliable results or conclusions.

**Table 3:** Comparison of the summary results of the three models.

Datasets	Deep leaning MSE	SVR MSE	SAE-SVR MSE	Promoted (%)	Deep learning MAE	SVR MAE	SAE-SVR MAE	Promoted (%)
1EURUSD	2.7307*e* − 04	0.0026098	2.88*E*−04	−5.60	0.0122	0.0399	0.02234	−83.11
2GBPUSD	6.8046*e* − 04	0.0011528	6.09*E*−04	10.51	0.0193	0.0272	0.01169	39.43
3AUDUSD	2.3025*e* − 04	0.0003145	1.95*E* − 04	15.22	0.0113	0.0143	0.01012	10.44
4EURGBP	2.6657*e* − 04	0.0015129	2.51*E* − 04	5.72	0.0122	0.0307	0.01149	5.82
5USDCAD	1.3537*e* − 04	0.0022363	1.82*E* − 04	−34.15	0.0085	0.0332	0.00922	−8.47
6EURCAD	2.9867*e* − 04	0.0005757	1.44*E* − 04	51.94	0.0126	0.0189	0.00984	21.90
7GBPCAD	2.2838*e* − 04	0.0007986	2.40*E* − 04	−5.00	0.0167	0.0215	0.01808	−8.26
8AUDCAD	4.8400*e* − 04	0.00068021	1.57*E* − 04	67.65	0.0167	0.0198	0.01089	34.79
9EURAUD	1.3568*e* − 04	0.00024962	4.12*E* − 05	69.66	0.0084	0.0114	0.00513	38.93
10GBPAUD	2.1326*e* − 04	0.00062255	2.77*E* − 04	−29.73	0.0109	0.0191	0.01465	−34.40
11USDJPY	1.4181*e* − 04	0.00465398	2.12*E* − 04	−49.77	0.0088	0.0567	0.01577	−79.20
12EURJPY	2.7442*e* − 04	0.00034466	7.06*E* − 05	74.29	0.0120	0.0142	0.00655	45.42
13GBPJPY	1.9389*e* − 04	0.00141236	9.14*E* − 05	58.26	0.1299	0.0299	0.0082	93.69
14CADJPY	4.2757*e* − 04	0.00055366	1.70*E* − 04	60.21	0.0149	0.0177	0.00939	36.98
15AUDJPY	3.6397*e* − 04	0.0002919	5.06*E* − 05	86.11	0.0136	0.0129	0.0089	34.56
16USDCHF	2.8011*e* − 04	0.0009669	3.42*E* − 05	87.80	0.0101	0.0154	0.00788	21.98
17EURCHF	1.9228*e* − 04	0.0022557	7.01*E* − 05	63.56	0.0061	0.0304	0.0049	19.67
18GBPCHF	3.0714*e* − 04	0.0010526	9.99*E* − 05	67.46	0.0103	0.0155	0.00541	47.48
19CADCHF	2.9759*e* − 04	0.00111476	4.82*E* − 05	83.81	0.0107	0.0208	0.00978	8.60
20AUDCHF	4.1407*e* − 04	0.0015979	9.80*E* − 05	76.33	0.0129	0.0268	0.01181	5.45
21CHFJPY	2.2217*e* − 04	0.0014423	4.14*E* − 05	81.35	0.0086	0.0224	0.00835	2.91
22USDCNY	8.7996*e* − 05	0.00103769	3.11*E* − 04	−253.22	0.0061	0.0135	0.0099	−62.30
23EURCNY	2.2732*e* − 04	0.0017301	2.94*E* − 04	−29.22	0.0110	0.0318	0.01578	−43.45
24GBPCNY	4.5092*e* − 04	0.00052641	1.68*E* − 04	62.79	0.0149	0.0163	0.01114	25.23
25CADCNY	1.7722*e* − 04	0.0045405	3.20*E* − 04	−80.78	0.0097	0.0536	0.01675	−72.68
26AUDCNY	2.3929*e* − 04	0.00255696	3.63*E* − 4	−51.88	0.0118	0.0403	0.01772	−50.17
27JPYCNY	1.9699*e* − 04	0.00255696	1.32*E* − 04	33.10	0.0099	0.0349	0.00086	91.31
28CHFCNY	0.0187	0.0316333	1.92*E* − 05	99.90	0.0886	0.1728	0.00438	95.06
Sum	—	—	—	610.92	—	—	—	240.61

The article "Exchange Rate Forecasting Based on Deep Learning and NSGA-II Models" was retracted in 2023. Reasons: signs of a paper mill; compromised peer review; unreliable results or conclusions.

## Data Availability

Relevant data are available upon request to all authors.
